# Text-Based Emotion Recognition Using Deep Learning Approach

**DOI:** 10.1155/2022/2645381

**Published:** 2022-08-23

**Authors:** Santosh Kumar Bharti, S Varadhaganapathy, Rajeev Kumar Gupta, Prashant Kumar Shukla, Mohamed Bouye, Simon Karanja Hingaa, Amena Mahmoud

**Affiliations:** ^1^Pandit Deendayal Energy University, Gandhinagar, India; ^2^Department of Information Technology, Kongu Engineering College, Erode, Tamil Nadu, India; ^3^Pandit Deendayal Energy University, Gandhinagar, India; ^4^Department of Computer Science and Engineering, Koneru Lakshmaiah Education Foundation, Vaddeswaram, Guntur, Andhra Pradesh, India; ^5^Department of Mathematics, College of Science, King Khalid University, Abha, Saudi Arabia; ^6^Department of Electrical and Electronic Engineering, Technical University of Mombasa, Mombasa, Kenya; ^7^Computer Science Department, Faculty of Computers and Information, Kafrelsheikh University, Kafr el-Sheikh, Egypt

## Abstract

Sentiment analysis is a method to identify people's attitudes, sentiments, and emotions towards a given goal, such as people, activities, organizations, services, subjects, and products. Emotion detection is a subset of sentiment analysis as it predicts the unique emotion rather than just stating positive, negative, or neutral. In recent times, many researchers have already worked on speech and facial expressions for emotion recognition. However, emotion detection in text is a tedious task as cues are missing, unlike in speech, such as tonal stress, facial expression, pitch, etc. To identify emotions from text, several methods have been proposed in the past using natural language processing (NLP) techniques: the keyword approach, the lexicon-based approach, and the machine learning approach. However, there were some limitations with keyword- and lexicon-based approaches as they focus on semantic relations. In this article, we have proposed a hybrid (machine learning + deep learning) model to identify emotions in text. Convolutional neural network (CNN) and Bi-GRU were exploited as deep learning techniques. Support vector machine is used as a machine learning approach. The performance of the proposed approach is evaluated using a combination of three different types of datasets, namely, sentences, tweets, and dialogs, and it attains an accuracy of 80.11%.

## 1. Introduction

In 1950, the birth of AI brought a significant change to the world. In the 20th century, AI is reintroduced in a bigger way and it brought researchers to do in-depth research in various fields such as NLP, computer vision, machine learning, and deep learning. However, the fields of NLP remain unclear due to its computational and linguistic techniques, which help computers understand and generate human-computer interactions in the form of text and speech. It aims at designing the model for different processes like perception, sentiment, beliefs, and emotions. Sentiment analysis finds out the sentiment of the given text in terms of positive, negative, or neutral. However, emotion analysis goes beyond that, which comes into effect by distributing the types under the sentiment analysis. Keyword-based and lexical affinity have been used to some extent because their drawbacks pull them down and give poorer accuracy than the learning-based approach. Machine learning and deep learning approaches are different in that they classify emotions in different ways. In this research, we have combined the datasets of 3 different types, namely, sentences, tweets, and dialogs, so that we can get a taste of 3 different variations. All the sentences were in the raw form, so for the better use of text sentences, we have preprocessed the data. Then put the data in different types of ML and DL models.

According to Ekman [1], emotions are categorized into 6 different types, as follows: joy, sadness, fear, surprise, anger, and disgust. Further, emotion is also described in various forms, such as love, optimism, etc., as shown in Figure 1 [2]. Facial expressions, gestures, speech, and text generally express the mood and emotions of a human being. Unlike facial expression and speech recognition, a text sentence loses the ability to define itself because it is tasteless. Because of the complexity and ambiguity of the text, it is a difficult task to find out the emotions of that text. It becomes a difficult task to recognize the emotion of a given text as each word can have a different meaning and morphological form.

In recent times, researchers have proposed various methods to detect the emotions of the text, such as keyword-based, lexical affinity, learning-based, and hybrid models [3]. In the beginning, they introduced a rule-based approach that consisted of two approaches, namely, lexical affinity-based and keyword-based. Later on, a new approach came into existence, i.e., the learning-based approach. This method was more accurate and gave better results. In a learning-based approach, different models are used to detect emotion. Many researchers have also started combining the approaches and making them hybrid in the search for high accuracy. As per the study, deep learning models show better accuracy than machine learning models for large sizes of text or data. But for small data, machine learning gives us better accuracy. Still, none of the approaches gave a complete solution to detect the emotion from a given text.

There were many limitations in the existing solutions, such as that they did not have a list of all the emotions. The existing lists have an inadequate vocabulary of words in the lexicon, disregarded words, semantics-based context, low extractions of contextual information from the given sentences, do not perform well for detecting some specific emotions; weak context information extraction, loose semantic feature extraction, less computational speed, ignored relations between features, an inadequate amount of data, and a high number of misclassifications. Some models were not suited well for frequently occurring emojis, weak semantic information extraction, and the structure of the sentence. It differs from model to model. There were many limitations in this system that were fulfilled by previous researchers. The proposed model has fulfilled many of the existing limitations.

Emotion detection is one of the big advantages of human-machine interaction as a nonliving thing can sense or feel like a human being. Our proposed model can detect emotions from text sentences that are tasteless as they do not have any tone or expression. Many researchers have worked on a single dataset. But we have worked on three datasets which include the textual form of simple sentences, tweets, and dialogs to detect emotions. Our text-based emotion recognition model can be implemented on any system. For business potential, this model can help to find emotions from customer reviews, services, give security for social media users, and many others.

The rest of the article is organized as follows: Section 2 presents the literature survey on emotion detection. The proposed scheme is explained in Section 3.  Section 4 draws results and analysis of the proposed work. Finally, Section 5 concludes the article with future directions.

## 2. Literature Review

Several studies have used various techniques to detect emotions from text [3–7]. It will show that which is the best model and gives us a higher accuracy.

Seal et al. [4] have performed emotion detection with a keyword-based approach mainly focused on phrasal verbs. They used ISEAR [5] data, preprocessed the data, and then applied the keyword-based approach. They discovered several phrasal verbs that should have been associated with emotion terms but were not, and so they built their own database. They recognized phrasal verbs and keywords synonymous with various emotions and categorized them using their database. They did, however, achieve a much higher accuracy of 65%, but they were unable to address the researcher's existing issues, such as an insufficient list of emotion keywords and a lack of respect for word semantics in meaning. The work by Alotaibi [7] has worked on a learning-based approach. He has used the ISEAR [5] database for emotion detection. Then, using classifiers like Logistic Regression, K-Nearest Neighbour (KNN), XG-Boost, and Support Vector Machine (SVM), he preprocessed and trained the data. According to him, all other classifiers poorly performed as compared to Logistic Regression. Finally, he said that the deep learning technique would help to improve the model.

Xu et al. [8] P. Xu et al. [12] has proposed an Emo2Vec method that encodes emotional semantics into vector form. They have trained Emo2Vec on a multitask learning framework by using smaller and larger datasets (smaller datasets such as ISEAR, WASSA, and Olympic). It shows that their results are better than those of Convolution Neural Network (CNN), DeepMoji embedding, and more. They have utilized their work on emotion analysis, sarcasm classification, stress detection, etc. Finally, the model Emo2Vec, when combined with Logistic Regression and GloVe, can achieve more competitive results. Ragheb et al. [9] W. Ragheb et al. [13]worked on detecting emotions from textual conversations through the help of learning-based model. Their data comprises 6 types of emotions that Paul Ekman has [1] described. In their methods, two phases of encoder and classification are present. After the data is collected, it is tokenized and passed to an encoder, which then passes it on to Bi-LSTM units that have been trained using average stochastic gradient descent (ASGD). To avoid over-fitting, they have applied dropouts between the LSTM units. Then, to focus on specific emotion-carrying conversations, a self-attention mechanism was used. The data was classified into its respective categories through the help of a dense layer and a SoftMax activation. The model showed an F1 score of 75.82%.

Suhasini and Srinivasu [10] M. Suhasini and B. Srinivasu [14]used a learning-based approach in which machine learning classifiers were used to detect or classify emotions. They have used KNN and Naive Bayes (NB) for the detection of emotions using tweets in the Sentiment 140 corpus. They compared the accuracy of the NB to that of the KNN, finding that the NB was 72.06% compared to the KNN's accuracy of 55.50%. The model's drawbacks are that they have low extractions of contextual information in the given sentences. Hasan et al. [11] M. Hasan et al. [15] used the supervised machine learning method and an emotion dictionary in their proposed model for recognizing emotions from the text. To carry out emotion classification, they performed two tasks, first offline and then online. Through the help of emotion-labeled text from Twitter and other classifiers, an offline model was developed for emotion classification. The training dataset was built by preprocessing the data. Then, the online approach classified streaming content of tweets in real time using the model developed in the offline approach [12]. Their model had a 90% overall accuracy.

Rodriguez et al. [13] use emotion analysis to identify hate speech on social media. Their aim with this research was to locate and analyse the unstructured data of selected social media posts that intend to spread hate in the comment sections. Cao et al. [14] exploited machine and deep learning approaches to evaluate emotion in textual data. They also highlight the issues and challenges regarding emotion detection in text. Acheampong et al. [15] F. A. Acheampong [20] surveyed the concept of emotion detection (ED) from texts and highlighted the main approaches adopted by researchers in the design of text-based ED systems. Navarrete Verma [16] P. Nandwani and R. Verma [21] described the process used to create an emotion lexicon enriched with the emotional intensity of words and focused on improving the emotion analysis process in texts [13]. Sailunaza and Alhajj [17] K. Sailunaz and R. Alhajj [22] used Twitter data to detect emotion and sentiment from text. They exploited sentiment and emotion scores to generate generalized and personalized recommendations for users based on their Twitter activity [4].

## 3. Proposed Scheme

This section describes the proposed system that consists of data collection and data preprocessing. After preprocessing, the data will move forward as an input to both ML and DL models. In ML, the preprocessed data will be given as the input to ML classifiers and will show the results of all ML classifiers. Furthermore, it will select the best ML model that gives the highest accuracy. In DL, the data is converted into vector form and given as an input to the DL models. Before that, we used a pretrained word vector to make the word embedding matrix and add the embedded layer to the DL model [18]. After performing on individual models, we combine the two best DL models based on accuracy and F1 score. Combining them will give us the latent vector and it will be given as an input to the best ML model for the prediction of emotions. Finally, it will select the best accuracy of all the ML, DL, and hybrid models. The pipelined diagram of our proposed model is shown in Figure 2.

### 3.1. Dataset Description

The data is taken from three different datasets: ISEAR, WASSA, and Emotion-stimulus, which have text and emotions as the attributes. These datasets consist of three different types of text: normal sentences, tweets, and dialogs.

The International Survey on Emotion Antecedents and Reactions (ISEAR) database [5] was built over a number of years in the 1990s by a vast community of psychologists from all over the world under the direction of Wallbott and Scherer. They experienced 7 types of emotions (joy, anger, guilt, sadness, disgust, fear, and shame). According to a cross-cultural survey conducted in 37 countries across five continents, as many as 3000 individuals from a wide range of backgrounds came together to discuss and debate the events.

The dataset is built on both emotional stimuli and statements [6]. The data was created for 173 emotions but grouped into 7 types of emotions (fear, sadness, anger, joy, disgust, surprise, and shame). The emotion “cause” dataset contains 820 sentences with both an emotion cause and a tag. And the no “cause” dataset contains 1594 sentences with only an emotion tag [5]. The description of the dataset is illustrated in Table 1.

In this research, all three data sets, namely, text sentences, dialogs, and tweets, are combined. The combined dataset contains over 14500 text sentences. Every text sentence is labeled with 6 forms of emotions as joy, disgust, fear, surprise, anger, and sadness (according to its syntactic and semantic polarities) [19]. These emotions are highlighted in Figure 3. The text is in English and has some additional punctuation and emojis with it. The dataset contains only text sentences and their corresponding emotions. Each dataset is divided into two types of data: training and testing, and the ratio is 80 : 20.

### 3.2. Data Preprocessing

The data is in raw form and must be preprocessed to eliminate unnecessary text and symbols. It is a data mining technique for converting raw data into a useable and effective format [20]. It boosts the efficiency of ML and DL models while conserving computational power. Many types of preprocessing tools are present according to our data. We have processed with the following: tokenization, stop words removal, emoji conversion to text, stemming, and lemmatization. In this research, we have used Natural Language Toolkit (NLTK) tools for all the preprocessing steps namely, tokenization, lemmatization, stop word removal, etc. The data is transformed from one format to another to make it easier to read and understand. Integrate the data since it comes from multiple sources and must be integrated before it is processed further [21]. The data gathered during the reduction process is nuanced, and it must be formatted to provide more precise results. The data is grouped and separated into training and testing datasets, and then run through different ML and DL algorithms to enhance the performance.

In this article, datasets are collected from three different sources, namely ISEAR, WASSA, and Emotion-stimulus. We need to preprocess the data to reduce the computational resources. For data preprocessing, we used a data cleaning method for the removal of noisy data from the text sentences [22]. Noisy data is considered as unwanted data for further processing, such as unnecessary text and symbols. These cleaned smooth sentences are then tokenized and given as input to the models.

### 3.3. Feature Extraction

It is a dimensionality reduction technique that reduce a large collection of raw data into smaller categories for faster processing [23].

#### 3.3.1. TF-IDF

The TF-IDF is a combined vector of term frequency and inverse document frequency. It identifies the most frequent terms within the document and rarely used terms across the document. It helps to choose a unique term vector as a feature set for training.

In this article, the TF-IDF Vectorizer transforms text to feature vectors so it can be used as input to an estimator. A vocabulary of a dictionary that converts each token (word) to a feature index based on their frequency in the matrix, and every unique token gets a feature index using

(1) $$\begin{array}{c} W\left(d,t\right)=TF\left(d,t\right)*\text{log }\left(\frac{N}{\text{d}f\left(t\right)}\right), \end{array}$$

where *d* represents documents, *t* represents terms in the document, and N denotes the total number of documents.

#### 3.3.2. Word Embedding's

In word embedding, there are four methods, namely, word2vec, Global vectors for word representation (GloVe), Embedding from Language Models (ELMO), and fast text. Among these methods, we have used wor2vec in our model. The word2vec algorithm learns word associations from a large corpus using a neural network model [15].

After preprocessing the dataset, we convert them into vector form. As we have different lengths of text sentences, the model will not handle the data, and we have to apply padding to each text [24]. The majority of the text has a length of 50. So, through the help of padding, small-sized text sentences are converted to the size of 50. By using a pretrained vector, we have built a matrix of (18210, 300).

### 3.4. ML  and  DL Models

These models are a form of artificial intelligence (AI) that helps a machine learn and evolve without being explicitly programmed [16]. The preprocessed training dataset is then given as input into the CountVectorizer, TF-IDF Transformer, and MLClassifier to train the model and predict the emotions on the test dataset.

This research used the prebuilt models of ML and DL. For ML, classifiers like DT, SVM, NB, and RF were built to predict emotions, and for deep learning, we deployed Gated Recurrent Unit (GRU), Bidirectional Gated Recurrent Unit (Bi-GRU), and Convolutional Neural Network (CNN) to predict emotions. All the ML and DL models are shown in Figures 4–7.

#### 3.4.1. Gated Recurrent Unit (GRU)

It helps to solve the vanishing gradient problem that a standard recurrent neural network (RNN) encounters [17]. Since both are constructed alike and, in some cases, yield equally excellent performance, the GRU may be considered a variant of the LSTM. The GRU model is a single layer in our proposed model. After feature extraction, the embedding layer of size (18210, 300) will be input for the GRU model shown in Figure 5. The training vector will be used as an input to the GRU model to predict the emotions for the data.

#### 3.4.2. Bidirectional Gated Recurrent Unit (Bi-GRU)

A Bidirectional GRU [25] is a sequence processing paradigm made up of two GRUs working together. One provides feedback in a forward direction, and the other in a backward direction. Just the input and output gates are used in this bidirectional recurrent neural network. The Bi-GRU model is a single layer in our proposed model. After feature extraction, the embedding layer of size (18210, 300) will be input for the Bi-GRU model shown in Figure 6. The training vector will be given as an input into the Bi-GRU model to predict the emotions for the data.

#### 3.4.3. Convolutional Neural Network (CNN)

It is a form of deep neural network used to analyse visual imagery in deep learning [26]. The CNN model is of a single layer in our proposed model. After feature extraction, the embedding layer of size (18210, 300) will be input for the CNN model shown in Figure 7. The training vector will be input into the CNN model to predict the emotions for the data [27].

### 3.5. Hybrid Model

The proposed hybrid model combines deep learning and machine learning algorithms to predict emotions. The overall system diagram is shown in Figure 8. Deep learning consists of CNN and Bi-GRU, and machine learning consists of an SVM classifier. It starts with input datasets, which are fed into the word embedding layer, i.e., word2vec. After getting the embedding vector, it needs to be fed into both the deep learning algorithms, namely, CNN and Bi-GRU. From CNN and Bi-GRU models, we have removed the last layer, and so they will act as encoders [28].

Furthermore, both of these encoders will generate a latent vector for the given input embedding vector. Lastly, these latent vectors will be concatenated and will be fed to the SVM classifier. The SVM classifier will predict the emotion of these input texts.

The proposed hybrid model gives improved results in terms of accuracy and F1 score due to the selection of classification models in both deep learning and machine learning. In the individual results of deep learning models, CNN and Bi-GRU performed well. Similarly, in the machine learning algorithms, SVM performed well [29]. Therefore, we choose the best classifiers from both categories to improve the result. In the hybrid model, we combined the ML and DL models, as shown in Figure 8. So, we combined the two best deep learning models, which give the best accuracy and F1 score. After getting the best DL models, the latent vector was given as an input to the best ML models, which predicts emotions as it shows high accuracy [30].

## 4. Results and Discussion

We have performed many experiments using various methods to get the best accuracy for our proposed model. Emotion classification with a machine learning approach, a deep learning approach, and our hybrid model approach on the multitext dataset consisting of sentences, tweets, and dialogs. Three datasets are used for performing these experiments.

First, the text was given as an input to the pipeline, which then converts text into a vector. These vectors were used to train the ML Classifier. The accuracy which is listed in Table 2 is from the machine learning approach.

Second, the features were extracted using the pretrained word vector, and the embedding matrix of size (18210, 300) was the input layer for the DL model. The padded vector was trained on the DL model.  Table 3 shows the accuracy of the DL models.

Finally, our hybrid model is a combination of both ML and DL models. Both the DL model CNN and Bi-GRU are combined, and the latent vector from them is an input vector for the SVM model for training the data.  Table 4 represents the accuracy of our proposed hybrid model.

As with the basic model of ML and DL, we get better results, but they are not the best results. The ML approach will give the best accuracy for different types of emotions, and the same for the DL approach. So, by combining the models, we get the highest accuracy.

Emotion detection from text is one of the most challenging and important tasks as it does not have any expression of emotions and the structure of text sentences. Researchers are trying hard to get a complete solution in this field, but they all have failed. But they have found the best solution for facial emotion expression and speech emotion recognition. Still, there is a mystery in this field.

## 5. Conclusion and Future Direction

In this paper, proposed a text-based emotion recognition model. The proposed model is a combination of deep learning and machine learning approaches. This proposed hybrid approach uses the combination of three datasets, namely, ISEAR, WASSA, and the Emotion-Stimulus dataset. The proposed model has many advantages, as it can work on multitext sentences, tweets, dialogs, keywords, and lexicon words of emotions that can be easily detected. According to the ML classifier, SVM gives the highest accuracy of 78.97%. In the DL method, the Bi-GRU model achieves the highest accuracy of 79.46%, and the CNN model achieves the highest F1-score of 80.76. The hybrid model has achieved a precision of 82.39, a recall of 80.40, an F1 score of 81.27, and an accuracy of 80.11%.

In the future, we will try more potential classifiers or ensemble techniques to improve the results. In the deep learning approach, we may get the combination of CNN, Bi-GRU, and LSTM to improve the results. Additionally, we will work on the structure of text sentences and some of the regional languages. Moreover, in this digital world, people's usage of sending text messages, uploading tweets, and writing online reviews of products have been in great use and demand. Therefore, by having a lot of data, we can make a real-time text-based emotion recognition model to find the emotions or moods of the people.

## Figures and Tables

**Figure 1:** Various types of Emotions.

**Figure 2:** Pipelined model of proposed scheme.

**Figure 3:** Six types of emotions in our Dataset.

**Figure 4:** Machine Learning model to detect emotions from text.

**Figure 5:** GRU model to detect emotions from text.

**Figure 6:** Bi-GRU model to detect emotions from Text.

**Figure 7:** CNN model to detect emotions from text.

**Figure 8:** Hybrid model to detect emotions from text.

**Table 1:** Individual description of all the datasets.

Dataset	Granularity	No. of emotions	Size	Description
ISEAR	Sentences	7 emotions	7666	Studied in 37 countries
WASSA	Tweets	4 emotions	4334	Tweets
Emotion-stimulus	Dialogs	7 emotions	2500	—

**Table 2:** Evaluation matrix for ML Classifiers

ML classifier	Precision	Recall	F1 score	Accuracy
SVM	**81.45**	**78.36**	**79.67**	**78.97**
RF	79.42	75.66	77.02	76.25
NB	61.75	51.41	49.61	68.94
DT	72.48	69.70	70.94	69.42

**Table 3:** Evaluation matrix for with DL model.

Deep learning	Precision	Recall	F1 score	Accuracy
GRU	78.37	78.94	78.65	78.02
Bi-GRU	80.62	79.64	80.09	**79.46**
CNN	**82.12**	**79.92**	**80.76**	79.32

**Table 4:** Evaluation matrix for our hybrid model.

Hybrid	Precision	Recall	F1 score	Accuracy
CNN + Bi-GRU + SVM	**82.39**	**80.40**	**81.27**	**80.11**

## Data Availability

The data that support the findings of this study are available on request from the corresponding author.
